RETRACTED

# Research on Recurrence Plot Feature Quantization Method Based on Image Texture Analysis

**DOI:** 10.1155/2022/2495024

**Published:** 2022-08-08

**Authors:** Yan Li, Zhan Li

**Affiliations:** ^1^School of Economics and Management, Dongguan University of Technology, Dongguan 523808, Guangdong, China; ^2^School of Business, Huaihua University, Huaihua 418000, Hunan, China

## Abstract

The nonlinear time-series analysis method, based on the recurrence plot theory, has received great attention from researchers and has been successfully used in multiple fields. However, traditional recurrence plots that use Heaviside step functions to determine the recursive behavior of a point in the phase space have two problems: (1) Heaviside step functions produce a rigid boundary, resulting in information loss; and (2) the selection of the critical distance, *ε*, is crucial; if the selection is inappropriate, it will result in a low-dimensional dynamics error, and as of now, there exists no unified method for selecting this parameter. With regard to the problems described above, the novelty of this article lies in the following: (1) when determining the state-phase point recursiveness, a Gaussian function is used to replace the Heaviside function, thereby solving the rigidity and binary value problems of the recursive analysis results caused by the Heaviside step function; and (2) texture analysis is performed on a recurrence plot, new ways of studying complex system dynamics features are proposed, and a system of complex system dynamic-like measurement methods is built.

## 1. Introduction

Recurrence is one of the most basic qualities of a dynamic complex system. Some similar behaviors possess similar approaches to development. This type of state recurrence phenomenon is called recursive behavior and indicates that at different points in time, complex systems possess similar dynamic behavior. Although recursive behavior in the natural world received interest relatively early on, it was limited by the computing technology of that time. Furthermore, higher-dimensional complex systems lacked effective processing methods and computing technology. Eckmann et al. [1] constructed a recurrence plot theory that provides a highly operable method for phase-space reconstruction and the analysis of complex systems. The intrinsic ideology behind this method is to construct a phase space that is equal to the state of a primary dynamic system by reconstructing a phase space, reverting to a high-dimensional evolution state of a one-dimensional time series, and reconstituting the one-dimensional sequence into the trajectory of the point in the high-dimensional phase space. On this basis, the dynamic laws and features of the evolution of the primary dynamic system can be further analyzed. The traditional analysis of a time series is usually carried out in the frequency domain or time domain, while chaotic time series have nonlinear features and are difficult to model and calculate with traditional methods. Therefore, the analysis of chaotic time series is usually carried out in phase space. In recent years, the recurrence plot method has gradually developed into an effective tool for analyzing chaotic time series. The theoretical basis of the recurrence plot method is the time-delay embedding theory, which was proposed by Takens [2]. It is believed that as long as the embedding dimension is not less than twice the attractor dimension of the primary dynamic system, the reconstructed phase space and the phase space of the primary dynamic system will have topological equivalence. Therefore, a one-dimensional time series can be embedded into a topologically equivalent high-dimensional phase space through phase-space reconstruction, so that a trajectory of the state vector of the dynamic system in the mathematical-phase space can be obtained. However, in the process of reconstructing the phase space, the embedding dimension and time delay are two important parameters. Although the delayed embedding theory has obtained good results in theory, in practical applications, this conclusion cannot be used to determine the embedding dimension. In practical applications, the false nearest neighbor method, constructed by Kantz [3], or the Cao algorithm [4–6], is used more often to calculate the embedding dimension of the system. For determining the time delay, *τ*, autocorrelation analysis is often used [7–10]. However, some scholars believe that the two parameters of embedding dimension and time delay are related, so they should be solved jointly. Kim et al. [11] were the first to try to comprehensively consider the joint determination method of the embedding dimension and delay time. Based on this idea, Tao et al. [12] further constructed a C-C method that uses a correlation integral to determine the values of the two parameters.

RETRACTED

Marwan et al. [13] and Runqiang and Zhu [14] proposed that the recurrence plot method is a nonlinear analysis method for reconstructing the recursive behavior of complex dynamic systems, which allows the phase-space manifold of complex dynamic systems to be studied intuitively. Lv et al. [15] posited that the recurrence plot method is a nonlinear dynamic analysis method based on the phase-space reconstruction theory, which can reflect the laws of the chaotic attractor of the original system. Pham [16] constructed a fuzzy recurrence plot, and the reproduction of the phase-space state can be visualized as a grayscale texture, which enhances the ability to analyze information patterns. The fuzzy recurrence plot method replaces the critical similarity threshold required by the traditional recurrence plot. Sipers et al. [17] constructed multilevel recurrence plots (MRPs) and pointed out that MRPs with only a few discretization levels can usually capture the attributes and shapes of signals more accurately than traditional RPS. Tamura and Ichimura [18] constructed a recurrence plot based on a MACD histogram for time-series classification and representation. Riedl et al. [19] analyzed the characteristics and application fields of generalized recurrence plots. In general, the nonlinear time-series analysis methods based on the recurrence plot theory have received much attention from researchers in various fields, and they have been successfully applied to many fields, such as geology [20–23], ecology and biology [24–26], neuroscience [27–31], economic dynamics [32–34], industrial manufacturing, mechanical damage, and monitoring [25, 35–40], medicine [41–44], image processing, and audio and video analysis [45–47]anda CNN-based magnetic fingerprinting system using recurrence plots (RPs) was proposed as sequence fingerprints. Ref. [48] investigated the state transitions in different brain regions locally using a univariate measure based on dynamical system analysis named the recurrence plot (RP).

In the traditional recurrence plot method, with regard to how to judge whether the phase point of the two states in the phase space is recursive, the selection of the critical distance, *ε*, is important, but it is also a difficult task. Selecting inappropriate parameters will cause the low-dimensionality dynamic error. However, there is no uniform method for selecting this parameter at present, so it is usually necessary for the researcher to select an appropriate method according to the actual situation to determine it. If the *ε* selected is too small, there may be no or few recursion points in the recurrence plot, resulting in the inability to observe the recursive features of the system; but if the *ε* selected is too large, it may appear that almost every point has recursive behavior with neighboring points, which will cause thick and long diagonal lines in the recurrence plot. The general principle is that *ε* should not exceed 10% of the standard deviation of the time series [22, 49]. In many scholars' studies of specific problems, the more common approach has been to set the threshold to a certain proportion of the variance or standard deviation of the time-series data to be analyzed. Zhong et al. [50] used the recurrence plot method to study EHG signals, and the threshold was selected to be 0.5 to 1 time the standard deviation of the EHG sequence. When Chen et al. [51] studied the HRY signal, the threshold was selected to be 12% of the standard deviation of the original sequence data. In the study of protein structure prediction by Yang et al. [52], the rule for determining the threshold was to observe the change in the recursion rate. When the recursive rate changes for the first time, the corresponding threshold is the one that is sought. In general, the selection of *ε* does not form a unified method. The determination method is closely related to the specific problem to be studied and has a certain degree of experience. This is also a major problem when using the recurrence plot method. For different research objects, there are usually large differences in the criteria for selecting *ε*, but there is a slight difference in the selection of *ε*, and the obtained recurrence plots will have large differences, which poses greater challenges to the stability and reliability of the research results. Especially when constructing a recurrence plot through phase-space reconstruction, the Heaviside step function is usually used to judge the recursive behavior of the phase point of the state. When the distance between the phase points of the two states in the phase space is less than *ε*, we think of these two states as appearing recursive and vice versa; these two states do not appear to have recursive behavior. These processing methods have two problems as follows. (1) The research results have a strong dependence on the selection of the critical distance *ε*, but currently, there is no universal method for the selection of *ε*. This is also a difficult problem that we currency face in the research of nonlinear time series using phase-space reconstruction and recurrence plot methods. (2) The Heaviside step function has a rigid boundary problem, which will cause the loss of the original complex system dynamic behavior information contained in the nonlinear time series. When a phase point of a state is exactly outside the hypersphere with a certain phase point as the center and *ε* as the radius, the two state-phase points are considered completely dissimilar, and the phase points of the states distributed in the hypersphere are considered to be completely similar, but the differences between the phase points of these states are ignored. The innovation of this article is as follows: the use of the Heaviside step function will cause the recursive analysis results to be rigid and binary, making the research results unreliable and thus increasing the difficulty of selecting *ε*. A slight change in *ε* or a change in the length and position of the time series will cause significant change to the results. In order to overcome the rigid boundary problem caused by the Heaviside step function, this article proposes using the Gaussian function instead of the Heaviside function when judging the recursiveness of the state-phase point. The Gaussian function can more accurately measure the recursive features of the two state-phase points in the reconstructed high-dimensional space. At the same time, as the Gaussian function has no rigid boundary, the recursiveness between all of the state-phase points in the reconstructed phase space can be determined by the state-phase distance between the points and the Gaussian function value. When the distance between the phase points of the state is 0, the degree of recursion between the phase points is 1; when the distance between the phase points of the state increases from zero to infinity, the degree of recursion between the phase points gradually changes from 1 to 0.

RETRACTED

## 2. Gaussian Function Recurrence Plot and Texture Features' Analysis

### 2.1. Gaussian Function Recurrence Plot

According to the time-delay embedding theorem, the phase-space reconstruction method can be used for the one-dimensional time series {*x*_*i*_ | *i* = 1,2,…, *n*}. By selecting the appropriate phase-space dimension, *m*, and the delay time, *τ*, the one-dimensional time series can be reconstructed into an *m*-dimensional phase space, at which point a state vector set, $R^{m}=\left\{\overset{⟶}{X_{i}}\right\}$, can be obtained, where $\overset{⟶}{X_{i}}=\left(x_{i},x_{i+\tau },\ldots ,x_{i+\left(m-1\right)\tau }\right),\;i=1,2,\ldots ,n^{*}$ and *n*^*∗*^ = *n* − (*m* − 1)*τ*. The vector set $\left\{\overset{⟶}{X_{i}}\;|\;i=1,2,\ldots ,n^{*}\right\}$ can be used to represent the state trajectory of a one-dimensional time series, {*x*_*i*_ | *i* = 1,2,…, *n*}, in a high-dimensional phase space. When the distance between the two state vectors in the phase space is less than *ε*, it can be considered that the two states exhibit recursive behavior of state recurrence. $R_{ij}=\Theta \left(\varepsilon -\overset{⟶}{X_{i}}-\overset{⟶}{X_{j}}\right),\;\overset{⟶}{X_{i}},\overset{⟶}{X_{j}}\in R^{m},\;i,j\in \left(1,2,\ldots ,n^{*}\right)$ and Θ(•) are Heaviside functions, and the values of $\Theta \left(x\right)=\left\{\begin{array}{c} 1,x\geq 0\\ 0,x<0 \end{array}\right.$ and *R*_*ij*_ represent the recursive relationship between the state vectors $\overset{⟶}{X_{i}}$ and $\overset{⟶}{X_{j}}$ in the phase space. All of the *R*_*ij*_ will form a matrix *R* of 0 s and 1 s, which is called a recursive matrix. The recursive matrix can be represented by a two-dimensional graph. The value “1” is represented by a black dot, which means that the state of the system at time *i* is reproduced at time *j*; the value “0” is represented by a white dot, which means that the state of the system at time *i* is not reproduced at time *j*. The recurrence plot can be obtained from the recurrence relationship between the state vectors at each point in time of the system. In addition to the embedding dimension and time delay, the selection of *ε* is also important. If different *ε* values are selected, different recursive graphs may be obtained. However, there is currently no universal method for selecting *ε*. At the same time, Heaviside step functions have a rigid boundary problem, which will cause the loss of the originally complex system information contained in the nonlinear time series. This article uses a Gaussian function instead of Heaviside step function, as Gaussian functions can take continuous values, and there is no rigidity problem; at the same time, the obtained Gaussian function value is expressed in different grayscale levels, from small to large. The state recursive features of the complex system in the phase space will show different texture features in the recurrence plot. By studying these texture features, the similarity, mutation, and dynamic evolution of the dynamic features of the complex system can be identified:

(1) $$\begin{array}{c} R_{ij}=e^{-\sum_{k=1}^{m}\left|X_{ik}-Y_{jk}\right|/s*\tau }, \end{array}$$

where *s* is the standard deviation of the time series {*x*_*i*_ | *i* = 1,2,…, *n*}, *m* is the embedding dimension, and *τ* is the time delay. When the state vectors $\overset{⟶}{X_{i}}$ and $\overset{⟶}{X_{j}}$ get close, *R*_*ij*_ approaches 1, and when the state vectors $\overset{⟶}{X_{i}}$ and $\overset{⟶}{X_{j}}$ grow further apart, *R*_*ij*_ approaches 0. In this way, a recursive matrix composed of numbers between 0 and 1 can be obtained. The larger the value of *R*_*ij*_, the darker the color, and vice versa. The sine signal sin(6*∗π∗t*) is constructed below, the sampling frequency is 1000 Hz, and 2000 data points are collected. The Lorentz signal has *σ* = 10,  *b* = 8/3,  *r* = 28, and the initial values of the three quantities are the time series generated by the *x* (*t*) component in the case of (12, 2, 9), the traditional recurrence plot, and the Gaussian function recurrence plot of a random time series [see Figure1].

RETRACTED

### 2.2. Recurrence Plot Texture Feature Similarity Analysis

#### 2.2.1. Texture Feature Extraction

The local binary pattern (LBP), proposed by Ojala et al. [53], is an operator used to extract local texture features of an image. It has significant advantages such as rotation invariance and grayscale invariance. The basic idea of the LBP algorithm is as follows: in a 3 *∗* 3 window, take the grayscale value of the central pixel of the window as a threshold and compare the grayscale value of the pixels of the adjacent 8 points with it. If the central pixel value is less than the surrounding pixel value, the position of the surrounding pixel is marked as 0; otherwise, it is 1. Using 8 points in the 3 *∗* 3 neighborhood with this operation, you can obtain an 8-bit binary number (usually converted to a decimal number; that is, in the LBP code, there are 256 types). In this way, the LBP value of the center pixel of the window can be obtained. Then, this value is used to reflect the texture features in this area. The basic operation is shown in Figure 2.

The formula to calculate the LBP code is

(2) $$\begin{array}{c} \text{LBP}\left(x_{c},y_{c}\right)=\sum_{n=0}^{p-1}2^{n}\Theta \left(i_{n}-i_{c}\right), \end{array}$$

where (*x*_*c*_, *y*_*c*_) is the center pixel; *i*_*c*_ is the grayscale value of the center pixel; *i*_*n*_ is the grayscale value of the neighboring pixels; and Θ(•) is the Heaviside function, where $\Theta \left(x\right)=\left\{\begin{array}{c} 1,x\geq 0\\ 0,x<0 \end{array}\right.$.

Using the LBP operator, an LBP “code” can be proposed for each pixel, and the normalized statistical histogram from the LBP code can reflect the texture feature information of the image. It can be seen from Figure 3 that the statistical histograms of the LBP code of the periodic time series, the chaotic time series, and the random time series are significantly different from each other, thus indicating that the systems that generate these time series have different dynamic behavior features. This shows that the statistical histogram of the LBP code can reflect the difference between the dynamic features of the complex system.

One of the shortcomings of the LBP coding statistical histogram is that the overall LBP coding is statistically analyzed. The distinguishing effect is not ideal in some cases. At this time, we can introduce the method of image block processing, which divides the image into several sub-blocks. For example, we can decompose the overall recurrence plot into *m∗n* subregions and perform LBP processing on this small *m* × *n* region separately. This can greatly enhance the analysis effect of the dynamic features of the complex system.

#### 2.2.2. Texture Feature Similarity Measure

Rubner et al. [54] constructed a method for measuring the similarity of image textures: Earth mover's distance (EMD). The basic idea of EMD is to precisely convert one type of distribution to the minimum cost that must be paid for another distribution. At first, the concept of EMD was mainly used for image retrieval work, and then, it was gradually used to measure similarity in other aspects. The EMD distance is actually the following linear programming problem. Suppose *P*={(*p*_1_, *w*_*p*1_), (*p*_2_, *w*_*p*2_),…, (*p*_*m*_, *w*_*pm*_)}, where *p*_*i*_ represents a feature of an image, and *w*_*pi*_ represents the weight of the feature *p*_*i*_. *Q*={(*q*, *w*_*q*1_), (*q*, *w*_*q*2_),…, (*q*, *w*_*qn*_)}, where *q*_*j*_ represents a feature of another image, and *w*_*pi*_ represents the weight of the feature *q*_*j*_. *D*=[*d*_*ij*_] represents the distance matrix of the difference between the feature *p* set and the feature *q* set, where *d*_*ij*_ represents the distance of features *p*_*i*_ and *q*_*j*_. Solve the matrix *F*=[*f*_*ij*_], where *f*_*ij*_ represents the amount of change from feature *p*_*i*_ to feature *q*_*j*_, and *d*_*ij*_ represents the cost (distance) of features *p*_*i*_ and *q*_*j*_. The goal is to minimize the global cost function:

(3) $$\begin{array}{c} \text{WORK}\left(P,Q,F\right)=\sum_{i=1}^{m}\sum_{j=1}^{n}f_{ij}d_{ij}. \end{array}$$

The following constraints must be met:

(4) $$\begin{array}{c} f_{ij}\geq 01\leq i\leq m,1\leq j\leq n,\\ \sum_{i=1}^{n}f_{ij}\leq w_{pi}1\leq i\leq m,\\ \sum_{i=1}^{m}f_{ij}\leq w_{pj}1\leq j\leq n,\\ \sum_{i=1}^{m}\sum_{j=1}^{n}f_{ij}=\min\left(\sum_{i=1}^{m}w_{pi},\sum_{j=1}^{n}w_{qj}\right). \end{array}$$

The first constraint indicates the change from *P* to *Q*; this cannot be reversed. The second constraint indicates that the total sum out of the amount of *p*_*i*_ cannot exceed the total amount *w*_*pi*_ of features *p*_*i*_. The third constraint indicates that the inflow of *q*_*j*_ cannot exceed the amount it can accommodate *w*_*qj*_. The fourth constraint indicates that the total amount of flow cannot exceed the total amount in *P* and the total amount that *Q* can accept. By solving this linear programming problem, we can get the optimal flow, *F*. To ensure that EMD does not change with the total flow, we can divide each flow by the total flow and normalize it. The distance between *P* and *Q* is

(5) $$\begin{array}{c} \text{EMD}\left(P,Q\right)=\frac{\sum_{i=1}^{m}\sum_{j=1}^{n}f_{ij}d_{ij}}{\sum_{i=1}^{m}\sum_{j=1}^{n}f_{ij}}. \end{array}$$

RETRACTED

## 3. Value Analysis

Logistic mapping is a simple one-dimensional dynamic system with extremely complex behavioral characteristics. It originated from the population model in ecology. The mapping can produce aperiodic and nonconvergent sequences. The difference equation for generating the logistic sequence is *X*_*n*+1_=*a∗X*_*n*_(1 − *X*_*n*_). *R*. May, a mathematical ecologist, published a classic paper in the journal Nature in 1976, and pointed out that when the parameter a changed within the interval [3.5, 4], the logistic map exhibited a period-doubling bifurcation leading to chaos. Later, after further research by Feigenbaum, it was concluded that if a system has a period-doubling bifurcation, it will inevitably lead to chaos. When the parameter a was closer to 4, the logistic sequence *X* was closer to the average distribution for all of 0 to 1. When a changed from 3.4 to 4.0, the step size was 0.0006, the initial value *X*_0_=0.512, and 2000 iterations were performed on each parameter value. After removing the first 1000 transient points, 1001 sequences could be obtained, and the graph *xa* was drawn, as shown in Figure 4. In Figure 4, at several vertical dotted lines (with parameter a as 3.4522, 3.5440, 3.5614, 3.6274, 3.6334, 3.7384, 3.7438, 3.8284, and 3.8464), the dynamic feature of logistic mapping exhibits substantial changes, and their performance in 10 different dynamic features regions is listed in the following order: 2 periods, 4 periods, 8 periods, chaos, 6 periods, chaos, 5 periods, chaos, 3 periods, and chaos. In order to further analyze the changes in the dynamic features of the logistic mapping on the corresponding parameter points, the following formula *λ*=(1/*N*)∑_*n*=1_^*N*^log_2_ was used to calculate the maximum Lyapunov exponent of the sequence obtained by the logistic mapping at each parameter point. The maximum Lyapunov exponent varies with the parameter a, as shown in Figure 5. When the Lyapunov exponent is less than 0, the region is a periodic region of logistic mapping, and if the reverse is true, the corresponding sequence is a chaotic sequence. It can be seen from Figure 5 that at the corresponding bifurcation point, the Lyapunov index exhibits a significant change.

When the Gaussian recurrence plot and its texture analysis method constructed in this article were used, it can be seen from Figure 6 that the Gaussian recurrence plot has clear texture differences at different parameter values, and the LBP coding statistical histogram also has significant differences.

Next, the method of measuring the similarity of the dynamic features of two complex systems constructed in the second part of this article was used to analyze the changes in the dynamic features of 1001 sequences obtained after removing the first 1000 transient points when parameter a changed from 3.4 to 4.0, with a step size of 0.0006 and *X*_0_=0.512, and each parameter value was subjected to 2000 iterations. A random sequence was used as a benchmark for comparison, and the similarity between each sequence and the random sequence is measured. The result is shown in Figure 7.

RETRACTED

When the parameter a is close to 4, after the parameter value a is determined, the initial value *X*_0_ has an impact on the time-series value generated by the entire system. The entire system exhibits chaotic phenomena, and even when the initial value changes little, the time series values obtained by the system show large differences. When the parameter *a*=3.99, the initial values are *X*_0_ = 0.663489000 and *X*_0_ = 0.663489001. At the beginning of the iteration, the difference between the two is small, approximately close 0, but as the number of iterations increases, the difference between the two sequences shows an irregularity. The magnitude of the change suddenly increases, so it can be seen that the system has a good avalanche effect, as shown in Figure 8(a). When we selected parameter *a* = 3.99, the initial value changed from 0.663489001 to 0.663489500, a total of 500 initial values were obtained, 2000 iterations were performed on each initial value, the first 1000 transient points were removed, and 500 time series were obtained. A random sequence was used as a benchmark for comparison to measure the similarity of dynamic features between each sequence and random sequence. The results are shown in Figure 8(b). Obviously, these sequences have the same dynamic feature similarity as random sequences.

## 4. Conclusion

In recent years, the recurrence plot method has gradually developed into an effective tool for analyzing chaotic time series. However, the traditional recurrence plot method uses the Heaviside step function to judge the recursive behavior of the state points in the phase space. The disadvantages of this processing method are that the results of the recursive analysis have rigidity and binary value problems. In order to overcome the rigid boundary problem caused by the Heaviside step function, this article proposes using the Gaussian function to replace the Heaviside function when judging the recursiveness of the state-phase point. At the same time, it puts forward the idea of texture analysis of recurrence plots with respect to the feature analysis of recurrence plots. On this basis, a method to measure the similarity of dynamic features of complex systems is constructed. Finally, a numerical analysis of the logistic system showed that the method constructed in this article could adequately describe the dynamic features of complex systems and measure the similarity of dynamic features between different complex systems. The method constructed in this article can provide an effective method for the feature extraction of complex system dynamics.

RETRACTED

## Figures and Tables

**Figure 1:** Traditional recurrence plot and recurrence plot of Gaussian function.

**Figure 2:** LBP code calculation.

**Figure 3:** LBP coding statistical histogram. (a) Sine sequence, (b) Lorenz sequence, and (c) random time sequence.

**Figure 4:** Logistic mapping sequence diagram.

**Figure 5:** Graph of the largest Lyapunov exponent.

**Figure 6:** Gaussian recurrence plot and LBP coding statistical histogram Gaussian. (a) Parameter *a* = 3.4438, (b) parameter *a* = 3.6730, (c) parameter *a* = 3.7168, (d) parameter *a* = 3.7162, (e) parameter *a* = 3.8296, and (f) parameter *a* = 3.9454.

**Figure 7:** Similarity between system dynamics features and stochastic system dynamics characteristics under various parameters.

**Figure 8:** Parameter *a* = 3.99, similarity of dynamic features under different initial values.

## Data Availability

No data were used to support this study.
